The article "A Fatal Case of Wernicke's Encephalopathy after Sleeve Gastrectomy for Morbid Obesity" was retracted in 2017. Reasons: errors in the results or conclusions; missing or withdrawn patient consent.

# A Fatal Case of Wernicke's Encephalopathy after Sleeve Gastrectomy for Morbid Obesity

**DOI:** 10.1155/2014/281210

**Published:** 2014-09-07

**Authors:** Dimitrios K. Manatakis, Nikolaos Georgopoulos

**Affiliations:** 2nd Surgical Department, Athens Naval and Veterans Hospital, 70 Deinokratous Street, Athens, Greece

## Abstract

Wernicke's encephalopathy is an acute neuropsychiatric disorder, due to thiamine (vitamin B1) deficiency. It is traditionally described in chronic alcohol abusers; however obesity surgery is an emerging cause, as the number of bariatric procedures increases. A high index of clinical suspicion is required, since initial symptoms may be nonspecific and the classic triad of ophthalmoplegia, gait and stance disorders, and mental confusion is present only in one-third of patients. Laboratory tests can be within normal range and typical MRI brain lesions are found only in 50% of cases. Aggressive supplementation with intravenous thiamine should not be delayed until confirmation of diagnosis, as it may fully reverse symptoms, but almost half the patients will still display permanent neurological deficit. We present our experience with a fatal case of Wernicke's encephalopathy, following laparoscopic sleeve gastrectomy for morbid obesity.

## 1. Introduction

As morbid obesity reaches alarming proportions in the West, the number of bariatric procedures steadily increases [1, 2]. Micronutrient deficiencies, long considered obsolete in developed countries, have reemerged and are an anticipated complication of malabsorptive bariatric surgery [2].

Restrictive procedures on the other hand are less prone to cause nutrient deficiencies, since the primary mechanism of action is reduction of food intake [3, 4]. We present our experience with a fatal case of Wernicke's encephalopathy (WE) due to thiamine deficiency, following laparoscopic sleeve gastrectomy for morbid obesity.

## 2. Case Presentation

A 51-year-old, male Caucasian patient underwent laparoscopic vertical sleeve gastrectomy for morbid obesity (BMI 41.5, comorbidity: diabetes mellitus II, sleep apnea, and social drinker). His early postoperative course was uneventful and he was discharged on the 6th postoperative day, after a gastrografin swallow test, which was negative for leakage.

Two months postoperatively and two weeks after resuming a normal diet, he was admitted in hospital with a 5-day history of protracted vomiting and malaise. Clinical examination revealed signs of dehydration. Laboratory tests (complete blood count, arterial blood gases, glucose, electrolytes, and kidney and liver function tests), plain abdominal radiographs, and abdominal CT scans were within normal range. Upper GI endoscopy was negative for sleeve stenosis and gastrografin swallow test revealed no delayed gastric emptying.

On the 5th day, he developed acute ophthalmoplegia with diplopia and weakness of the left arm. Brain CT and MRI scans showed no pathological findings of hemorrhagic or ischemic stroke and he was admitted in the department of neurology for further diagnostic workup. Lumbar puncture findings were within normal range; EEG showed no focal lesions and EMG revealed polyradiculoneuropathy. Neostigmine test was also negative. His clinical condition continued to deteriorate, with generalized muscle weakness, drowsiness, and confusion. Three days later he developed ileus, which was complicated with lower respiratory tract infection, possibly because of aspiration.

Despite parenteral nutrition and vitamin supplementation, his vitamin B1, B2, and C levels were low and diagnosis of WE secondary to thiamine malabsorption was established. High dose (500 mg tid) of thiamine supplementation was initiated; however the patient was intubated two days later, due to respiratory failure, and was transferred to the ICU, where he died three weeks later.

## 3. Discussion

Although most patients remain asymptomatic, micronutrient deficiencies are not uncommon after bariatric surgery. Postoperative deficiencies and supplementation requirements vary among procedures, depending on which segment of the gastrointestinal tract is affected [5]. Deficiencies may complicate any type of bariatric surgery but tend to occur more frequently after malabsorptive, rather than purely restrictive, procedures [3, 6–8].

WE is an acute neuropsychiatric disorder caused by thiamine (vitamin B1) deficiency. The disorder is traditionally described in chronic alcohol abusers but has also been associated with malnutrition, malabsorption, prolonged fasting or parenteral nutrition, gastrointestinal malignancies, dialysis, AIDS, and bariatric surgery [5, 8]. Limited, existing evidence suggests an incidence of 0.2% after malabsorptive procedures, but the incidence after restrictive procedures remains unknown [9]. A search of the English-speaking literature revealed only 8 cases of thiamine deficiency after sleeve gastrectomy and they are related to postoperative hyperemesis gravidarum, poor eating habits, or noncompliance of patients to dietary instructions [10–17]. As the number of postoperative WE cases rise, the term bariatric beriberi has emerged in the literature [9]. The actual size of the problem however may be underestimated, as indicated by autopsy studies [18].

Thiamine is a water-soluble vitamin, acting as coenzyme in carbohydrate metabolism. It functions as a cofactor of various enzymes, most importantly the *α*-ketoglutarate-dehydrogenase complex and the pyruvate-dehydrogenase complex in the tricarboxylic pathway and transketolase in the pentose-phosphate pathway [18].

It is found in pork, poultry, eggs, fish, legumes, nuts, and whole grains. Dairy products, fruits, and vegetables are not an adequate source [2]. Absorbed in the duodenum and proximal jejunum by active transport, it is converted to its active metabolite, thiamine pyrophosphate, after crossing the blood-brain-barrier [18].

Thiamine requirements are directly related to both total caloric intake and proportion of carbohydrate calories. Consequently, high energy and high carbohydrate diets increase demands in thiamine [18]. The recommended daily allowance in adults is 500 *μ*g per 1000 kilocalories but is higher in children, critically ill patients, during pregnancy and lactation, and after major surgery or trauma [2, 18]. Liver storage is adequate only for ~3 weeks, while tea and coffee contain thiaminase, an enzyme that breaks down ingested thiamine [2]. A possible genetic predisposition in individuals with reduced transketolase activity is also being investigated [5].

WE is clinically characterised by mental confusion, gait and stance ataxia, and ophthalmoplegia with nystagmus [5]. However the classic triad is only present in 16–38% of patients [9, 11]. Cases presenting with atypical symptoms have also been described; therefore a high index of clinical suspicion is required in patients with prior history of bariatric surgery, unbalanced diet, and progressing neurological symptoms [5, 7, 8].

There is no specific routine laboratory test for the diagnosis of WE [18]. Cerebrospinal fluid tests, electroencephalogram, and evoked potentials can all be within normal range [18]. Serum thiamine concentration and red blood cell transketolase activity could confirm clinical suspicion, but they are technically difficult, time-consuming, and neither widespread nor readily available [8, 9, 18].

Brain computed tomography has limited potential in differentiating pathological findings lesions. Magnetic resonance imaging is currently considered the most valuable option, with typical lesions in 50% of patients [9, 19]. These include symmetric hyperintensity on T2-weighted and FLAIR images; symmetric hypointensity or no abnormalities on T1-weighted images; and symmetric contrast enhancement after gadolinium injection in the thalamus, periventricular region of the third ventricle, mamillary bodies, periaqueductal area, tectal region, and periventricular gray matter of the fourth ventricle [19, 20]. Although MRI has a specificity of 93%, a sensitivity of 53% means that a normal scan cannot exclude the diagnosis of WE [19]. Moreover, recent evidence suggests that MRI findings may differ among nonalcoholic and alcoholic patients, with brain areas considered atypical for the disease affected more frequently in the former [20].

As early symptoms may be vague and nonspecific, initial working diagnosis is usually that of stroke [21]. Timely recognition of affected patients can be difficult but is of utmost importance, since intense supplementation of thiamine may fully reverse symptoms. Dramatic improvement with thiamine administration practically confirms the diagnosis [11].

The optimal treatment regimen is still a matter of debate, but thiamine supplementation should be aggressive [9]. Most authors agree on a dosage scheme of 500 mg of intravenous thiamine three times daily for 2-3 days, followed by 250 mg i.v. daily until improvement [5, 18]. Under no circumstances should thiamine administration be delayed until diagnosis is confirmed [9]. Delay in treatment leads inadvertently to permanent neurological deficits or death [5–9, 18]. However, even with replacement therapy, almost half the patients will still exhibit permanent cognitive impairment, as shown in a review of 84 confirmed cases of postbariatric surgery WE [9, 21].

Prevention is therefore the best strategy. Patients should be thoroughly instructed as to proper dietary habits. It is also crucial to explain the risks of excessive vomiting and rapid weight loss [9]. Prophylactic thiamine should be initiated to patients readmitted after bariatric surgery and those reporting protracted vomiting, even in the absence of symptoms [9].

Follow-up laboratory tests and micronutrient supplementation instructions vary greatly among bariatric surgeons, as does patient compliance with the recommended regimens [3, 4]. The updated Clinical Practice Guidelines for the Perioperative Nutritional, Metabolic and Nonsurgical Support of the Bariatric Surgery Patient, published in 2013 by the American Association of Clinical Endocrinologists (AACE), The Obesity Society (TOS), and the American Society for Metabolic and Bariatric Surgery (ASMBS), state that “*Thiamine supplementation should be included as part of routine multivitamin with mineral preparation (Grade D). Routine thiamine screening is not recommended following bariatric surgery (Grade C; BEL 3). Screening for thiamine deficiency and/or empiric thiamine supplementation should be considered in postbariatric surgery patients with rapid weight loss, protracted vomiting, parenteral nutrition, excessive alcohol use, neuropathy or encephalopathy, or heart failure (Grade D)*” [1].

Interestingly there is a growing body of evidence to suggest that obese individuals display a higher prevalence of micronutrient deficiencies than normal-weight individuals, due to poor quality of food intake (“high-calorie malnutrition”) [2, 7, 22]. A review by Kaidar-Person et al., evaluating morbidly obese patients, reported an incidence of 15–29% of preoperative thiamine deficiency [2]. In their studies, Ernst et al. and Gehrer et al. found that one in two patients (48.5% and 57% resp.) had at least one subnormal parameter at the preoperative assessment, with the most frequent deficiencies involving vitamins D, B12, and zinc [7, 22]. These studies emphasize the need for preoperative assessment and supplementation of vitamins and minerals in obese patients before surgical treatment.

## 4. Conclusion

This case report once more illustrates the need for a multidisciplinary team in treating morbid obesity. Despite hi-tech imaging and expensive blood tests, WE remains a clinical diagnosis. Surgeons may not be familiar with the clinical presentation of micronutrient deficiencies, resulting in unnecessary delay in diagnosis and treatment. In hyperemetic patients with deteriorating neurological status and history of bariatric surgery, a high index of suspicion and a low threshold for aggressive supplementation with intravenous thiamine are mandated. Therapeutic administration of thiamine should not be delayed, while waiting for confirmation of diagnosis with laboratory and imaging tests, as this may prove catastrophic.
